The article "Analysis on the Application Effect of Abdominal Acupoint Massage on Feeding Intolerance in Premature Infants" was published in 2021. Journal: J Healthc Eng.

# Analysis on the Application Effect of Abdominal Acupoint Massage on Feeding Intolerance in Premature Infants

**DOI:** 10.1155/2021/2883597

**Published:** 2021-12-02

**Authors:** Li Zhu, Yueqiu Gong

**Affiliations:** Department of Pediatrics, Suzhou Hospital of Traditional Chinese and Western Medicine, Suzhou 215101, Jiangsu, China

## Abstract

**Objective:**

Breast milk is the best food for newly born infants because it is more digestible and can relieve infants' gastrointestinal burdens. The purpose of this study was to investigate the application effect of abdominal acupoint massage on feeding intolerance in premature infants.

**Methods:**

A total of 50 premature infants with feeding intolerance admitted to our hospital from January 2018 to October 2019 were selected and randomly divided into the control group (*n* = 25) and the experimental group (*n* = 25). Among them, the premature infants in the control group received routine therapy, while based on the treatment in the control group, the premature infants in the experimental group were treated with abdominal acupoint massage. After that, the incidence of feeding intolerance, MNA nutritional status score, body mass, development state, length of hospital stay, and response rate were all compared between the two groups to analyze the application effect of abdominal acupoint massage on feeding intolerance in premature infants.

**Results:**

The incidence of feeding intolerance of the premature infants in the experimental group was significantly lower than that in the control group, with statistically significant differences (*P* < 0.05); the MNA nutritional status scores of the premature infants in the experimental group were significantly higher than those in the control group, with statistically significant differences (*P* < 0.05); the body mass and development state of the premature infants in the experimental group were significantly better than those in the control group, with statistically significant differences (*P* < 0.05); the length of hospital stay of the premature infants in the experimental group was significantly shorter than that in the control group, with statistically significant differences (*P* < 0.05); the response rate in the experimental group was significantly higher than that in the control group, with statistically significant differences (*P* < 0.05).

**Conclusions:**

Abdominal acupoint massage therapy can significantly reduce the incidence of feeding intolerance, shorten the length of hospital stay, and improve nutritional status, development state, and response rate in premature infants, with obvious therapeutic effect, which is worthy of application and promotion in clinical practice.

## 1. Introduction

Without full-term birth, premature infants are prone to malnutrition, maldevelopment, and other health problems, compared with fetuses born at term [1–3]. Generally, breast milk is more digestible and can relieve infants' gastrointestinal burdens; besides, breast milk contains some immune factors, which can effectively prevent immune diseases in infants. Premature infants have immature digestive system physiological functions and gastrointestinal neuroendocrine regulation, especially premature infants with a small gestational age and low body weight at birth. They have weak gastrointestinal motility and lack the motivation to advance food. Feeding intolerance can cause a series of short-term and long-term adverse effects. However, quite a few premature infants easily suffer from feeding intolerance, which is mainly manifested by gastric retention, abdominal distension, etc., and lack attention to this disease which may lead to severe gastrointestinal diseases in infants [3–5]. The leading causes of feeding intolerance include congenital gastrointestinal diseases, dysphagia, and sucking disorders, and there have been so many studies on analyzing the causes of feeding intolerance in premature infants, which also come with a variety of solutions [6, 7]. Studies have shown that oral massage can significantly relieve feeding intolerance and reduce adverse reactions that occur with feeding in premature infants, and other reports have also revealed that infantile massage can alleviate feeding intolerance and promote the growth and development in premature infants. Acupoint massage is one of the most commonly used therapies in traditional Chinese medicine with a total of 720 acupoints in the human body, including 402 acupoints commonly used [8–10], and the role of each acupoint in the human body is different; therefore, acupoint massage should be performed specifically according to patients' own conditions. At present, there are just few studies on the application effect of abdominal acupoint massage therapy on feeding intolerance in premature infants. Kai and Xiang [11] scholars pointed out that infantile massage can obviously alleviate feeding intolerance and adverse reactions in premature infants, which is in line with the findings of our study that abdominal acupoint massage therapy can significantly relieve feeding intolerance in preterm infants, demonstrating the reliability of our study results. Based on this, in this study, in order to investigate the application value of abdominal acupoint massage therapy on feeding intolerance in premature infants, premature infants with feeding intolerance were selected as the study subjects to analyze the therapeutic effect of different therapies on feeding intolerance. Specific studies are reported as follows.

## 2. Materials and Methods

### 2.1. General Information

A total of 50 premature infants with feeding intolerance admitted to our hospital from January 2018 to October 2019 were selected and randomly divided into the control group (*n* = 25) and the experimental group (*n* = 25). There were no statistically significant differences in general information such as preterm birth time and birth time between the two groups (*P* > 0.05), as shown in Table 1.

### 2.2. Inclusion/Exclusion Criteria

#### 2.2.1. Inclusion Criteria

- Premature infants had the gestational age of less than or equal to 38 weeks
- Premature infants had the birth time of less than or equal to 1 month
- Premature infants had no congenital diseases and no familial hereditary diseases
- Premature infants had no respiratory diseases and no circulation system diseases
- This study was approved by the Hospital Ethics Committee, and the families of premature infants all voluntarily participated in this study and signed informed consent

#### 2.2.2. Exclusion Criteria

- Premature infants were delivered at term
- Premature infants were twin or multiple preterm births
- Premature infants had organic diseases

### 2.3. Methods

The premature infants in the control group were treated with routine therapy in which the premature infants were mainly fed with breast milk according to the rules of small amount and high frequency after being guided to suck on their own. After that, medical staff should press infants' abdomen; auxiliary exhaust should be performed if infants had significant abdominal distension, and corresponding treatment methods should be carried out once infants had vomiting or defecation difficulties. In addition, premature infants should be given bifid triple viable capsules dissolving at intestines (manufacturer: Jincheng Hais Pharmaceutical Co., Ltd; State Food and Drug Administration approval no. S19993065; specification: 0.21 g ∗ 36 capsules) for oral administration, with one capsule at a time, twice a day, and for 7 consecutive days in total.

Based on the therapy in the control group, the premature infants in the experimental group were given abdominal acupoint massage therapy by massaging abdominal Yin and Yang acupoints for 5 min each on both sides and kneading Zhongwan acupoint clockwise and counterclockwise for 5 min each, 3 times a day, and the massage should be performed at 1 hour after the meal and continued for 1 course of 1 month.

### 2.4. Observation Indexes

The incidence of feeding intolerance, MNA nutritional status score, body mass, development state, length of hospital stay, and response rate were all compared between the two groups.

Feeding intolerance referred to gastric retention, abdominal distension, vomiting, defecation difficulties, etc., in premature infants during being fed.

With MNA nutritional status score ranging from 0 to 30 points, the score of more than 23.5 points indicated good nutritional status, the score of 17–23.5 points indicated moderate malnutrition, and the score of less than 17 points indicated severe malnutrition [12–14].

Response rate was categorized into the markedly effective, effective, and ineffective. No occurrence of feeding intolerance during feeding indicated the markedly effective, the condition that mild intolerance such as abdominal distension occurred but it disappeared after massage indicated the effective, and the condition that severe intolerance with vomiting occurred and gastric tube feeding was in need indicated the ineffective.

### 2.5. Statistical Treatment

Data processing software selected in this study was SPSS 20.0, and GraphPad Prism 7 (GraphPad Software, San Diego, USA) was used to draw the pictures of the data. Measurement data were expressed by ($\bar{x}$ ± *s*) and tested by *t*-test. Enumeration data were expressed as *n* (%) and tested by *X*^2^ test. The differences had statistical significance when *P* < 0.05.

## 3. Results

### 3.1. Comparison of the Incidence of Feeding Intolerance of the Premature Infants between the Two Groups

After different therapies for premature infants in both groups were performed for 1 month, the incidence of feeding intolerance in both groups was compared, and the results showed that the premature infants in the experimental group only had slight abdominal distension after feeding, and the symptoms relieved significantly after massage, while the premature infants in the control group still had gastric retention, abdominal distension, and vomiting. The incidence of the feeding intolerance in the experimental group was significantly lower than that in the control group, with statistically significant differences (*P* < 0.05), indicating that abdominal acupoint massage therapy can reduce the incidence of feeding intolerance and relieve the adverse reactions of the premature infants, as shown in Table 2.

### 3.2. Comparison of the MNA Nutritional Status Score between the Two Groups

The MNA nutritional status score of the premature infants in the experimental group was significantly higher than that in the control group, with statistically significant differences (*P* < 0.05), suggesting that abdominal acupoint massage therapy can obviously improve malnutrition in premature infants and promote nutrition absorption, as shown in Figure 1.

### 3.3. Comparison of the Body Mass and Development State of the Premature Infants between the Two Groups

After 1 month of treatment, the results showed that the changes of body mass and development state of the premature infants in the experimental group were significantly higher than those in the control group, with statistical significance (*P* < 0.05), indicating that abdominal acupoint massage therapy can promote growth and development in preterm infants, as shown in Table 3.

### 3.4. Comparison of the Length of Hospital Stay of the Premature Infants between the Two Groups

The length of hospital stay of the premature infants in the two groups can reflect the therapeutic effect, and a shorter length of hospital stay indicated better therapeutic effect. Study results showed that the length of hospital stay of the premature infants in the experimental group was significantly shorter than that in the control group, with statistical significance (*P* < 0.05), as shown in Figure 2.

### 3.5. Comparison of the Response Rate between the Two Groups

The response rate of the premature infants in the experimental group was 88%, which was significantly higher than that of 60% in the control group, with statistical significance (*P* < 0.05), suggesting that the application of abdominal acupoint massage therapy for premature infants with feeding intolerance can significantly relieve feeding intolerance and improve response rate, as shown in Table 4.

## 4. Discussion

402 acupoints include dead acupoints which can lead to patients' death after being severely hit, so the implementation of acupoint massage should be guided by professional doctors [15–17]. Feeding intolerance is a common disease affecting newborn infants, which is mainly manifested by gastric retention, abdominal distension, and other symptoms caused by dyspepsia after being fed. Intolerance occurs because the functions of various organs have not fully developed in newborn infants, who cannot digest food in a timely manner after feeding. In general, the best food for newborn infants is breast milk, but feeding intolerance often occurs when some parturients cannot provide breast milk for some reasons such as breast milk insufficiency or suffering from infectious diseases [18–21]. In addition, compared with the fetuses delivered at term, premature infants have more incomplete development of various functions and a larger incidence of feeding intolerance. Some studies have reported that massage can significantly improve feeding intolerance. In this study, the premature infants with feeding intolerance were selected, and they were treated with different therapies; the premature infants in the control group received routine therapy, while based on the treatment in the control group, the premature infants in the experimental group were treated with abdominal acupoint massage. After that, the application effect of abdominal acupoint massage on feeding intolerance in premature infants was analyzed.

The findings indicated that preterm infants in the experimental group had greatly improved their feeding intolerance after receiving abdominal acupoint massage therapy for 1 month, and the incidence of feeding intolerance in the experimental group was significantly lower than that in the control group, with statistical significance (*P* < 0.05), indicating that abdominal acupoint therapy significantly reduces the incidence of feeding intolerance and relieves adverse reactions in premature infants during being fed.

Moreover, the comparison of the nutritional status and development state of the premature infants between the two groups after 1-month treatment indicated that the nutritional status and development state of the preterm infants in the experimental group were significantly better than those in the control group, with statistical significance (*P* < 0.05), suggesting that abdominal acupoint massage can promote nutrition absorption in premature infants and avoid malnutrition. Additionally, the comparison of the length of hospital stay between the two groups revealed that the length of hospital stay in the experimental group was significantly shorter than that in the control group, with statistical significance (*P* < 0.05), showing that abdominal acupoint massage therapy can significantly reduce the length of hospital stay and reduce the financial pressure on family members of premature infants. The MNA nutritional status scores of the premature infants in the experimental group were significantly higher than those in the control group, with statistically significant differences (*P* < 0.05); the body mass and development state of the premature infants in the experimental group were significantly better than those in the control group, with statistically significant differences (*P* < 0.05); the length of hospital stay of the premature infants in the experimental group was significantly shorter than that in the control group, with statistically significant differences (*P* < 0.05); the response rate in the experimental group was significantly higher than that in the control group, with statistically significant differences (*P* < 0.05).

In conclusion, abdominal acupoint massage therapy can significantly reduce the incidence of feeding intolerance, improve nutritional status and development state, and shorten the length of hospital stay in premature infants, with high application value and obvious therapeutic effect, which is worthy of application and promotion in clinical practice.

## Figures and Tables

**Figure 1:** Comparison of the MNA nutritional status score between the two groups. Note: the abscissa represented the experimental group and control group, while the ordinate represented the MNA score. ^*∗*^The comparison of the MNA score between the experimental group of 25.26 ± 2.06 points and the control group of 20.14 ± 2.33 points, with statistical significance, *t* = 8.23, and *P* < 0.001.

**Figure 2:** Comparison of the length of hospital stay of the premature infants between the two groups. Note: the abscissa represented the experimental group and control group, while the ordinate represented the length of hospital stay (LOS, d). ^*∗*^The comparison of the length of hospital stay between the experimental group of 30.16 ± 3.54 d and the control group of 35.29 ± 4.08 d, with statistical significance, *t* = 4.75, and *P* < 0.001.

**Table 1:** Comparison of the general information between the two groups ($\bar{x}$ ± *s*).

Group	Experimental group	Control group	*t*/*X*^2^	*P*
Gestational age (weeks)	33.52 ± 2.04	33.90 ± 2.00	0.67	0.51
Birth time (d)	5.37 ± 1.66	5.41 ± 1.27	0.10	0.92
Body mass (kg)	2.88 ± 0.93	2.81 ± 0.99	0.26	0.80
Height (cm)	26.51 ± 6.24	26.38 ± 6.08	0.07	0.94
Gender (male/female)	13/12	14/11	0.08	0.78
First parturition (cases)	23	22	0.22	0.64
Family heredity history	0	0		
Congenital disease	0	0		

**Table 2:** Comparison of the incidence of feeding intolerance of the premature infants between the two groups.

Group	Gastric retention	Abdominal distension	Vomiting	Total incidence
Experimental group	0	4	0	16%
Control group	2	8	5	60%
*X* ^2^				10.27
*P*				0.001

**Table 3:** Comparison of the body mass and development state of the premature infants between the two groups ($\bar{x}$ ± *s*).

Group	Changes of body mass (kg)	Changes of height (cm)	Changes of head circumference (cm)
Experimental group	3.61 ± 1.03	5.57 ± 2.04	3.37 ± 0.48
Control group	1.39 ± 1.25	4.00 ± 1.37	1.28 ± 0.33
*T*	6.85	3.19	17.94
*P*	<0.001	0.003	<0.001

**Table 4:** Comparison of the response rate between the two groups.

Group	Markedly effective	Effective	Ineffective	Total response rate
Experimental group	16	6	3	88%
Control group	6	9	10	60%
*X* ^2^				5.09
*P*				0.02

## Data Availability

The datasets used and/or analyzed during the current study are available from the corresponding author upon reasonable request.
